This article has been retracted.

# Risk Factor Analysis of Hepatic Encephalopathy and the Establishment of Diagnostic Model

**DOI:** 10.1155/2022/3475325

**Published:** 2022-07-19

**Authors:** Fangfang Chen, Jing Li, Wenjie Zhang, Caixia Mao, Yanxia Wang, Yan Qu, Shuju Tian, Fanhong Li

**Affiliations:** Department of Hepatology, The Affiliated Hospital of Northwest University for Nationalities, The Second People's Hospital of Gansu Province, China

## Abstract

To identify laboratory diagnostic indicators of hepatic encephalopathy (HE), the present study established a HE diagnostic model to explore the diagnostic value of serum homocysteine, lactic acid, procalcitonin, and bile acid levels in HE identification. 371 patients with liver cirrhosis were selected as research objects, who were admitted to the Department of Hepatic Diseases, Affiliated Hospital of Northwest Minzu University from August 2019 to August 2020. The Spearman correlation results indicated that between lactic acid, procalcitonin, bile acid, serum homocysteine, and HE, the coefficients were -0.15, 0.41, 0.29, and -0.19, respectively. Univariate and multivariate analysis methods were adopted for inpatient analysis to identify the influencing factors of HE occurrence, and the diagnosis of the HE identification model was subsequently constructed. The univariate logistic regression showed that risk of developing HE increased as bile acid level (*P* = 0.00434) and serum homocysteine (*P* = 0.058) increased. Multivariate logistic regression diagnostic model of bile acid level and serum homocysteine revealed that the AUC value of the area under the ROC curve was 0.7201, indicating that the diagnostic model produced a satisfactory evaluation effect. The model formula referred logistic (*P*) = −2.4544 + 0.0117 bile acid levels + 0.0198 serum homocysteine. In this study, the HE diagnostic model was established using logistic regression analysis, which could benefit patients in early HE differential diagnosis. Particularly, combined detection of serum homocysteine and bile acid levels was considered to be more significant.

## 1. Introduction

Hepatic encephalopathy (HE) is a complex syndrome caused by liver disease, which is characterized by neurological, neuropsychiatric, and motor complications [1, 2]. It is prevalent in patients with acute, subchronic, and chronic liver failure as well as animal models. This disease is recognized as a common complication of severe liver disease and one cause of death. The latest research on the incidence of HE in China has stated that about 40% of hospitalized patients with liver cirrhosis developed minimal hepatic encephalopathy (MHE), while 30%-45% of cirrhosis patients and nearly 50% of patients with transjugular intrahepatic portal shunt surgery suffered from overt hepatic encephalopathy (OHE) [3, 4]. Current HE guidelines have pointed out that HE continuum covers a complete process from impaired cognitive function of the brain to conscious coma. HE is divided into covert hepatic encephalopathy (CHE) and OHE. The former includes MHE and grade 1 HE, and the latter contains grades 2, 3, and 4 HE. The main diagnosis of HE is the diagnosis of MHE and OHE. OHE is diagnosed based on clinical manifestations and physical signs and graded referring to the WeSt-Haven classification system [5, 6]. The procedures are not difficult, and basically, it needs no neuropsychological, neurophysiological, and imaging examinations. The present diagnosis of MHE is highly subjective with relatively difficulty in diagnosis and easy to be missed. MHE patients have higher potential risks, especially for drivers and those who work high above the ground. It is therefore that there is an urgent need for a simple and fast objective predictor to diagnose HE, especially for MHE patients [7–9].

Homocysteine is a nonprotein-forming amino acid that can activate ionotropic glutamate N-methyl-aspartate (NMDA) receptors, thereby causing Ca^2+^ to flow into neurons, which in turn activates several pathways, triggers oxidative stress, inflammation and apoptosis, and causes excitotoxicity [10]. Elevated levels of homocysteine in the plasma and brain develop hyperhomocysteinemia. Hyperhomocysteinemia activates NMDA receptor-mediated excitotoxicity and is related to a variety of diseases, including Parkinson's disease and Alzheimer's disease [11, 12]. Homocysteine is related to the occurrence of liver cirrhosis and related complications, but there is no relevant research on whether homocysteine is involved in the occurrence of HE [11]. In addition to neurotoxicity, inflammatory factors play an important role in the development of HE. Procalcitonin is a prototype of a hormone activating factor, which can be released from all cells in the body through microbial infection, but there is no current detailed information reported on the interrelationship between elevated procalcitonin and HE. Additionally, the pathogenesis of cerebral edema due to chronic liver failure is associated with elevated lactic acid including the factor of elevated glutamine. The increased lactic acid levels and the occurrence of HE may be related to the disorder of the brainstem reticulum system. Unfortunately, there are few studies on the risk of lactic acid and the occurrence of HE. Besides, the level of bile acid is also associated with HE cognitive and psychological abnormalities. The abnormal bile acid signaling pathway can activate nuclear receptor FXR, which may play a role in MHE development.

HE is currently diagnosed mainly based on the diagnosis of blood ammonia and the nervous system. However, it is relatively difficult for patients with CHE or OHE grade 1 or 2. This article is aimed at exploring the differentiation and diagnostic value of serum homocysteine, lactic acid, procalcitonin, and bile acid levels in HE.

## 2. Materials and Methods

### 2.1. Sample Information

This prospective study was conducted in the Department of Hepatic Diseases, Affiliated Hospital of Northwest Minzu University. The research selected patients with liver cirrhosis who were admitted to the Department of Hepatic Diseases, Affiliated Hospital of Northwest Minzu University, from August 2019 to August 2020, as research objects and investigated the incidence of HE and high-risk factors for the occurrence of HE in the selected population and determined the HE diagnosis model. This study was approved by the Ethics Committee of the Affiliated Hospital of Northwest Minzu University. Before starting each protocol-specific procedure, the informed consent of all participants have been obtained. This research was conducted following the principles in the Declaration of Helsinki (October 1983) [13].

### 2.2. Inclusion and Exclusion Criteria

Inclusion criteria are as follows: known cirrhosis and 18-70 years of age.

Exclusion criteria are as follows: other causes of ascites, including tuberculosis, spread of peritoneal cancer, appendicitis, pancreatitis, and hemorrhagic ascites and related causes of hyperhomocysteinemia including thrombosis, neuropsychiatric diseases, fractures, cancer, especially hepatocellular carcinoma, diabetes, heart failure, renal function impairment (serum creatinine > 1.8 mg/dl), thyroid hypofunction, and any type of infected cirrhotic patient other than spontaneous bacterial peritonitis (SBP).

### 2.3. Collection of Specimens

5 ml venous blood and 1 ml of EDTA whole blood were collected by venipuncture, and 4 ml of serum homocysteine without anticoagulation. Routine examinations were performed to analyze complete blood count, serum creatinine, total bilirubin, serum albumin, aspartate aminotransferase, alanine aminotransferase, prothrombin time, serum vitamin B6 determination, folic acid, vitamin B12, procalcitonin, total bile acid, lactic acid, and homocysteine.

### 2.4. Statistical Analysis

All statistical analysis adopted SPSS 23.0 (SPSS Inc., Chicago, Illinois, USA). The results were summarized as mean standard deviation. *χ*^2^ was used for comparison of distribution data. Paired *t*-test was applied to analyze the differences among each group. Spearman correlation analysis was also used. Receiver operating characteristic curve (ROC) and area under the curve (AUC) were both plotted to clarify the sensitivity and specificity of the model (*P* < 0.05 was considered statistically significant) [14].

## 3. Results

### 3.1. Spearman Correlation Analysis Was Adopted to Analyze the Correlation between Lactic Acid, Procalcitonin, Bile Acid, and Serum Homocysteine and HE

The information used in this study were obtained from 371 patients (227 males, 144 females), including 56 patients with hepatic encephalopathy (34 males, 22 females). After the Spearman correlation analysis between lactic acid, procalcitonin, bile acid, serum homocysteine ,and HE, the results were presented in Figure 1. The correlations between lactic acid, procalcitonin, bile acid, serum homocysteine, and HE were -0.15, 0.41, 0.29, and -0.19, respectively.

### 3.2. Results of the Univariate Logistic Regression Analysis

Subsequently, patients with hepatic encephalopathy were assigned a value of 1, and those with nonhepatic encephalopathy were assigned a value of 0; males were assigned a value of 1, and females were assigned a value of 0. Binomial logistic regression analysis was performed. The results as exhibited in Table 1 showed that the univariate logistic regression diagnosis model of bile acid level was significant (*P* = 0.00434), and OR > 1 indicated that the risk of developing HE increased as the bile acid level increased. The univariate logistic regression model of serum homocysteine was close to significant (*P* = 0.058), and OR > 1 indicated that the risk of developing HE increased as the serum homocysteine value increased. ROC curves were plotted using bile acid and serum homocysteine, respectively, and evaluated the significant univariate logistic regression diagnosis model based on the AUC values of the ROC curve. The AUC value of the ROC curve of the logistic regression model for bile acid levels was 0.83, the sensitivity was 0.715, and the specificity was 0.944. The AUC value of the ROC curve of the univariate logistic regression model for the serum homocysteine was 0.724, the sensitivity was 0.535, and the specificity was 0.913 (Figure 2).

### 3.3. HE Diagnosis Model Establishment Based on Multivariate Logistic Regression Analysis

Next, we included the four factors in the analysis and compared the results of the diagnostic model including the bile acid levels and serum homocysteine. The forest plot of the HE diagnosis model indicated that bile acid and serum homocysteine had a significant effect on HE (*P* < 0.05) (Figure 3(a)). The AUC value of the ROC curve was 0.7031, indicating that the multivariate logistic regression diagnostic model was accurate in diagnosis (Figure 3(b)). Both the previously described univariate and multivariate analysis results indicated the significance of bile acid levels and HE and close to significance of serum homocysteine and HE. It was therefore that both factors were selected to construct a multivariate logistic regression diagnostic model.

The diagnostic model forest plot of the multivariate logistic regression of bile acid levels and serum homocysteine was shown in Figure 3(c). The AUC value of the ROC curve the diagnostic model of the multivariate logistic regression for bile acid levels and serum homocysteine was 0.7201, indicating that the diagnostic model produced good performance for evaluation. The model formula was logistic (*P*) = −2.4544 + 0.0117 bile acid levels + 0.0198 serum homocysteine.

## 4. Discussion

Hepatic encephalopathy is a common complication of severe liver disease, which poses a threat to people's lives. It is an urgent need to develop a model for HE diagnosis [15]. This study recruited 371 patients with liver cirrhosis, including 56 HE cases. Based on univariate analysis, correlation analysis, and logistic regression analysis, it clarified that the levels of bile acid and serum homocysteine of patients were significantly correlated with HE, and finally, the HE diagnosis model was developed. The model formula referred logistic (*P*) = −2.4544 + 0.0117 bile acid levels + 0.0198 serum homocysteine. The present research offered certain novel ideas and references for the early diagnosis of HE.

Some recent studies have suggested that hyperhomocysteinemia as a result of abnormal hepatic homocysteine metabolism due to chronic liver disease (CLD) plays an important role in the occurrence and development of HE by activating NMDA receptors [16]. Hyperhomocysteinemia may act synergistically with hyperammonemia to activate NMDA receptors in the brain, resulting in oxidative stress, inflammation, apoptosis and neuron loss, thereby leading to HE [11]. Similarly, a prospective study has found that in rats with cirrhosis induced by common bile duct ligation, the improvement of hyperhomocysteinemia can substantially reduce both portal pressure and the risk of occurrence of CLD-related adverse events including HE and gastrointestinal bleeding [17, 18]. An additional study on SBP in CLD victims has found interrelationship between serum homocysteine and SBP, and the level of serum homocysteine serves as a predictor for CLD-SBP [19, 20]. Recently, high concentrations of bile acids have been found in the cerebrospinal fluid of patients with liver cirrhosis [21]. Studies performed in animal models have shown that rats with acute galactosamine liver failure develop focal cerebral edema, indicating that at least partial of the blood-brain barrier function is lost [22]. In the bile duct ligation (BDL) model, circulating bile acids increase significantly whereas the integrity of the blood-brain barrier decreases. According to the previously described studies, the increase in serum bile acid is not only a sign of biliary tract disease but also presents in ALF, ACLF, and nonalcoholic steatohepatitis [21]. Moreover, extravasation of bile acids has also been observed involving in circulation in the cerebrospinal fluid of patients with cirrhosis. It is therefore that a new understanding of the direct role of bilirubin or bile acid in the development of HE is necessary. In this study, Spearman correlation analysis was applied to analyze the correlation levels of bile acid and serum homocysteine and HE, which were 0.29 and -0.19, respectively. Multivariate logistic regression diagnostic model of bile acid level and serum homocysteine revealed that the AUC value of the ROC curve was 0.7201, indicating that the diagnostic model produced a satisfactory evaluation effect. The model formula referred logistic (*P*) = −2.4544 + 0.0117 bile acid levels + 0.0198 serum homocysteine.

When microorganisms in the body are infected, the host Toll-like receptor 4 (TLR4) can be activated and expressed in different immune cells, such as neutrophils, monocytes, macrophages, and dendritic cells, which generate inflammatory mediators and induce a variety of inflammatory processes [23, 24]. In the early inflammatory stage, procalcitonin is secreted by cytokine-activated macrophages and interacts with epithelial cells. In the postinflammatory stage, marked increase of IL-1*β* and TNF-*α* can induce the expression of procalcitonin. Furthermore, hepatocyte damage and inflammation may be the reason why the level of procalcitonin is positively correlated with the severity of liver disorders. Lactic acid is an organic molecule synthesized from glucose and metabolized by lactate dehydrogenase and presents in neurons and astrocytes. Lactic acid is transported to the extracellular space and used as an energy substrate by neurons. Traditionally, increased brain lactic acid is considered a sign of energy failure/injury, but recent research has indicated that lactic acid homeostasis alternation is related to neuronal dysfunction and HE. Some reports have pointed out that HE patients have elevated lactic acid concentrations in the systemic circulation and brain [25]. Experiments on BDL rats showed that the contents of lactic acid and glutamine in the brain increased with the increase of brain edema, while the inhibition of lactic acid synthesis reduced the lactic acid and brain edema in the brain and the increase in extracellular cerebral lactic acid correlated with the increase of intracranial pressure. This study included four factors for analysis. The results of forest plot of the HE diagnosis model revealed that bile acids and serum homocysteine had a significant impact on HE (*P* < 0.05), while procalcitonin and lactic acid did not act as a significant factor.

## 5. Conclusions

The logistic regression analysis demonstrated that serum homocysteine and bile acid levels was able to be employed for the establishment of the HE diagnostic model which can produce good performance for evaluation. The HE diagnostic model could benefit patients in early HE differential diagnosis.

## Figures and Tables

**Figure 1:** Univariate correlation analysis of lactic acid, procalcitonin, bile acid, serum homocysteine, and HE using the Spearman correlation analysis. Red represented positive correlation, and blue represented negative correlation. Larger absolute value indicated higher correlation.

**Figure 2:** ROC curves for bile acids and serum homocysteine, respectively.

**Figure 3:** Establishment of HE diagnosis model based on multivariate logistic regression analysis. (a) Forest plot analysis results after incorporating the four factors of lactic acid, procalcitonin, bile acid, and serum homocysteine. (b) Analysis results of ROC curve after incorporating the four factors of lactic acid, procalcitonin, bile acid, and serum homocysteine. (c) The diagnostic model forest plot of the multivariate logistic regression of bile acid levels and serum homocysteine. (d) ROC curve of the diagnostic model of multivariate logistic regression of bile acid levels and serum homocysteine.

**Table 1:** Results of the univariate logistic regression analysis.

	OR	OR_LCI	OR_UCI	*P*_value
Gender	0.98	0.55	1.75	0.937
Age	1.03	1	1.06	0.081
Lactic acid	0.84	0.59	1.2	0.339
Procalcitonin	1.03	0.96	1.11	0.367
Bile_acid_levels	1.01	1	1.02	0.00434
Serum_homocysteine	1.02	1	1.04	0.058

Remarks: OR: odds ratio; LCI: lower confidence interval; UCI: upper confidence interval.

## Data Availability

The data used to support the findings of this study are included within the article.

## References

[1] Mandiga P., Foris L. A., Bollu P. C. (2022). *Hepatic Encephalopathy. [Updated 2022 Mar 9]. In: StatPearls [Internet]*.

[2] Karanfilian B. V., Park T., Senatore F., Rustgi V. K. (2020). Minimal hepatic encephalopathy. *Clinics in Liver Disease*.

[3] Rustgi V. K. (2020). History of hepatic encephalopathy. *Clinics in Liver Disease*.

[4] Elsaid M. I., Rustgi V. K. (2020). Epidemiology of hepatic encephalopathy. *Clinics in Liver Disease*.

[5] Rodenbaugh D., Vo C. T., Redulla R., Mccauley K. (2020). Nursing management of hepatic encephalopathy. *Gastroenterology Nursing*.

[6] Jaffe A., Lim J. K., Jakab S. S. (2020). Pathophysiology of hepatic encephalopathy. *Clinics in Liver Disease*.

[7] Ryu A. J., Rahimi R. S., Leise M. D. (2020). The current hepatic encephalopathy pipeline. *Journal of Clinical and Experimental Hepatology*.

[8] Karanfilian B. V., Cheung M., Dellatore P., Park T., Rustgi V. K. (2020). Laboratory abnormalities of hepatic encephalopathy. *Clinics in Liver Disease*.

[9] Weiss N., Housset C., Thabut D. (2019). Hepatic encephalopathy: another brick in the wall. *Journal of Hepatology*.

[10] Czarnecka A. M., Hilgier W., Zielinska M. (2020). S-Adenosylmethionine deficiency and brain accumulation of S-adenosylhomocysteine in thioacetamide-induced acute liver failure. *Nutrients*.

[11] Choudhury S., Borah A. (2015). Activation of NMDA receptor by elevated homocysteine in chronic liver disease contributes to encephalopathy. *Medical Hypotheses*.

[12] Vakil A., Guru P., Reddy D. R., Iyer V. (2015). Diffuse cholangiocarcinoma presenting with hepatic failure and extensive portal and mesenteric vein thrombosis. *BML Case Reports*.

[13] Burlando M., Russo R., Clapasson A. (2020). The HLA-Cw6 dilemma: is it really an outcome predictor in psoriasis patients under biologic therapy? A monocentric retrospective analysis. *Journal of Clinical Medicine*.

[14] Almasri B., Ali A. (2021). Role of endoscopic ultrasound elastography in differential diagnosis of pancreatic solid masses. *Qatar Medical Journal*.

[15] Liere V., Sandhu G., Demorrow S. (2017). Recent advances in hepatic encephalopathy. *F1000Research*.

[16] Sim W. C., Yin H. Q., Choi H. S. (2015). L-serine supplementation attenuates alcoholic fatty liver by enhancing homocysteine metabolism in mice and rats. *The Journal of Nutrition*.

[17] Wu K. C., Huang H. C., Chang T. (2018). Effect of sirolimus on liver cirrhosis and hepatic encephalopathy of common bile duct-ligated rats. *European Journal of Pharmacology*.

[18] Gantzel R. H., Kjaer M. B., Laursen T. L. (2021). Macrophage activation markers, soluble CD163 and mannose receptor, in liver fibrosis. *Frontiers in Medicine*.

[19] Shaikh B. A., Shaikh Z. A., Shah A. H., Kumar A. (2021). Determining the risk of spontaneous bacterial peritonitis due to increase use of proton pump inhibitors among cirrhotic patients with ascites. *Pakistan Journal of Medical Sciences*.

[20] Garcia-Pagan J. C., Saffo S., Mandorfer M., Garcia-Tsao G. (2020). Where does TIPS fit in the management of patients with cirrhosis?. *JHEP Reports*.

[21] Hadjihambi A., Arias N., Sheikh M., Jalan R. (2018). Hepatic encephalopathy: a critical current review. *Hepatology International*.

[22] Quinn M., Mcmillin M., Galindo C., Frampton G., Pae H. Y., Demorrow S. (2014). Bile acids permeabilize the blood brain barrier after bile duct ligation in rats via Rac1-dependent mechanisms. *Digestive and Liver Disease*.

[23] Chen L. J., He J. T., Pan M. (2021). Antibiotics attenuate methamphetamine-induced hepatotoxicity by regulating oxidative stress and TLR4/MyD88/Traf6 axis. *Frontiers in Pharmacology*.

[24] Pires-Neto O. S., de Sa K. S., Santana B. B. (2015). Lack of association between polymorphisms of the TLR4 gene and Infection with the hepatitis B and C viruses. *Mediators of Inflammation*.

[25] Bosoi C. R., Rose C. F. (2014). Elevated cerebral lactate: implications in the pathogenesis of hepatic encephalopathy. *Metabolic Brain Disease*.

